The article "Blockchain Information Sharing Mechanism Based on Embedded System in Project Management System" was retracted in 2023. Reasons: signs of a paper mill; suspected computer-generated content; unreliable results or conclusions; concerns about the data.

# Blockchain Information Sharing Mechanism Based on Embedded System in Project Management System

**DOI:** 10.1155/2022/1835626

**Published:** 2022-08-04

**Authors:** Jinzhao Tian, Yisheng Liu, Meng Yang, Ruijiao Sun, Xiaoxiao Zheng

**Affiliations:** School of Economics and Management, Beijing Jiaotong University, Beijing 100044, China

## Abstract

As a new force for online reconstruction, blockchain will bring major changes to resource-sharing activities and information service organizations. The research introduces blockchain and related technologies, provides two basic ways of sharing data sources, and conducts two extensive information source sharing based on blockchain. The article analyzes the various challenges that need to be overcome to implement a blockchain-based information sharing system and suggests that project information service organizations should actively deal with the challenges brought about by blockchain. Experimental research is being conducted on a blockchain-based control system, and a blockchain-based blockchain management system is being developed. On the basis of system analysis and design, the most important functional components of the software system are developed. They include functions such as recording customers, logging in, storing information, printing device information, invoking server-side smart contracts, and conducting audit management. It uses decentralized payments and statistical aggregation of data. The experimental results show that the efficiency of using the blockchain information sharing mechanism in the management system is 35% higher than that of the traditional method, which can more effectively deal with the problem of information delay during the project management process.

## 1. Introduction

Construction project management involves the participation of construction units, survey and design, construction contracting, consulting and supervision units, and other subjects. With the increasing scale, complexity, and internationalization of construction projects, the exchange and transmission of information are becoming more and more frequent. The traditional information management mode and means cannot meet the needs of project management, and digitization has become the development trend of construction project management. As structured, information should be shared in an organized environment in some way and used appropriately, efficiently as well as fully. Information sharing is the foundation of the management field and an important goal of information retrieval, transmission, and processing, and therefore immediately became an area of interest. Through the development of social media and the rapid development of IT technology, in recent years, new strategies and new formats of technologies such as the Internet of Things, smart digital, big data, Internet+, and artificial intelligence have emerged. It affects the methods and functions of shared information systems. Taking advantage of the high-tech technological advancement in the real estate sector, blockchain is widely used in banking, securities, insurance, and other financial institutions, as well as in many fields. The development of the Internet and other companies in the past two years is a catalyst for future changes in the value of the Internet. It will also advance the way information is shared.

The article "Blockchain Information Sharing Mechanism Based on Embedded System in Project Management System" was retracted in 2023. Reasons: signs of a paper mill; suspected computer-generated content; unreliable results or conclusions; concerns about the data.

With the advancement of technology and application development, through the rapid promotion and dissemination of local needs, the rapid development and user participation of blockchain can be understood differently through the knowledge of each individual in the community. It has led to major changes in the creation of information sources, their distribution, intellectual property protection, and public access to information. It will also bring great changes to archives, documentation, and information service organizations. In the past decade, China's information technology industry has grown faster than it has in the same period. The amount of investment and the scale of construction in the information technology industry continue to increase. The proportion of the information industry in the gross national product has also increased to 12.5%, and the investment has reached 4 trillion yuan. The size of the market should not be underestimated, and it has gradually become a pillar industry in China's important industries. Enterprises are becoming more and more active in their demands for IT technology theory and application.

Blockchain originates from Bitcoin, a new payment system and a new digital currency. The blockchain is the underlying technology and infrastructure that supports Bitcoin. Blockchain is through distributed ledger technology (DLT), and it links a series of multiple blocks and records all data shared among each user in a network. These include peer-to-peer (P2P) technology and asymmetric encryption algorithms. Merkel encryption currency in data mining technology and tools hash algorithm timestamp technology, resolution, etc., are both new technologies created by increasing the knowledge of existing information technology or by combining existing information technology with alternative applications. While blockchain is based on Bitcoin, it is independent of Bitcoin for businesses. It can select or create different security systems. And the Bitcoin virtual currency can be interpreted differently. It is one of the growing Internet trends to have a complete awareness of blockchain-shared databases and shared scripts.

The article "Blockchain Information Sharing Mechanism Based on Embedded System in Project Management System" was retracted in 2023. Reasons: signs of a paper mill; suspected computer-generated content; unreliable results or conclusions; concerns about the data.

The remainder of this article is organized as follows: Section 2 is the related work.  Section 3 demonstrates the information sharing mechanism in project management. The experimental research process, results, and discussion can be found in Section 4 and Section 5. A comprehensive conclusion and future implementation of this research are in Section 6.

## 2. Related Work

Olnes et al. believed that as the technology behind Bitcoin, blockchain is an open distributed ledger. It records transactions securely, permanently, and efficiently [1]. The purpose of the Iansiti et al. study was to explore the application of blockchain technology in relation to the fourth industrial revolution and to show an example of using blockchain to facilitate machine-to-machine interaction and establish an M2M electricity market in China [2]. Dorri et al. believed that blockchain is a disruptive technology that has found many applications from cryptocurrencies to smart contracts. It is a potential solution to these challenges [3]. The central question discussed by Sikorski et al. was whether blockchain technology will lead to innovation and transformation of government processes. To address this issue, the benefits of blockchain technology, which are often exaggerated in the literature, have been critically assessed [4]. Zhou et al. proposed a contracting scheme based on prediction sharing. Under this scheme, GPOs can achieve perfect supply chain coordination in terms of quantity and information sharing. All members in the supply chain can achieve a win-win outcome [5]. Mansfield-Devine mentioned the word “blockchain” to most people. Assuming they have heard of it, they are likely to associate it with Bitcoin or another cryptocurrency. As a decentralized, cryptographically verified record of transactions, blockchain is the key concept that makes Bitcoin viable [6]. However, the above studies were not convinced by the public due to insufficient data.

## 3. Information Sharing in Project Management

It examines the project management information system from the perspective of knowledge generation, characteristics, distribution, and innovation, explains the source and content of project management information, and provides characteristics and distribution [7]. Project management knowledge and its corresponding transformation relationship provide a methodological theoretical basis for studying the composition and connection of project information management knowledge. According to the characteristics of project management, the information sharing characteristics of project management are analyzed. This framework provides a solution for research on sharing project management information [8].

The article "Blockchain Information Sharing Mechanism Based on Embedded System in Project Management System" was retracted in 2023. Reasons: signs of a paper mill; suspected computer-generated content; unreliable results or conclusions; concerns about the data.

It introduces the concept of collaboration to create an information platform for sharing storage and transportation resources through collaborative research. During the research process, the operating system takes blockchain as the core technology. It includes the user-centric application layer system technology, as well as the server-side TomCat server system. The blockchain takes the Ethereum utilities as the core platform. It intercepts the call through the interface, writes the user transaction information into the blockchain, and uses the blockchain to store the data at the end of the database [9]. On the basis of obtaining information sharing, it writes smart contracts for the warehousing and shipping process. It utilizes the implementation functions of the Ethereum operating system and antimonopoly blockchain technology, so that not all network maintenance orders can be exchanged [10]. Decentralized fixed payment solves the problem of a shared project management mechanism. The main research material of the article is its application in project management. The relationship is shown in Figure 1 [11, 12].

Shared information, same as cooperative consumption, expands infrastructure through full-capacity integration of products and services. Among them, the Oxford English Dictionary defines the economic sector as economically, the goods or services that people share through free or paid means [13]. Currently, as the Chinese economy changes and expands, economic participation has become a new model for future economic growth. According to the 2016 “China Sharing Economy Development Report,” China's economic growth in 2015 exceeded 195 million US dollars, accounting for 1.59% of GDP. Information is also spread out to meet different needs. In today's new economic environment, the sharing economy needs to use the integration of resources such as capital and information technology as a means, with the goal of improving resource utilization, and to realize the temporary transfer of resources [14]. It uses nonessential elements as the basis for the ability to establish the mutual aid relationship between supply and demand, rebuild the connection between the two, and understand the changes in the “supply side” and “demand side.” It effectively reduces the problem of information asymmetry between supply and demand and forms the exchange and sharing of the industrial ecological environment. Compared with the traditional economy, the top priority is the sharing platform and the other four elements that constitute the sharing economy. Suppliers are nonessential suppliers, and the rest needs to be distributed by both parties. A shared platform is a place to understand the role of sharing and build bridges of communication. Within the framework of understanding the sharing economy, sharing platforms seamlessly integrate infrastructure with network support. It establishes balance and listening between supply chain needs and demands, while building business trust through e-mail technical support that provides security features for the implementation of human resource development programs. The components of the shared platform are shown in Figure 2 [15, 16].

The article "Blockchain Information Sharing Mechanism Based on Embedded System in Project Management System" was retracted in 2023. Reasons: signs of a paper mill; suspected computer-generated content; unreliable results or conclusions; concerns about the data.

Information sharing has created a logistics model under the sharing economy. Due to the volatility of logistics itself, in order to ensure sufficient logistics resources to maintain normal operations, enterprises need to take effective measures to reduce logistics compliance [17, 18]. The emergence of shared information is to resolve differences caused by factors such as seasons, holidays, and environments, improve connectivity between systems, and avoid wasting resources. Shared logistics can be defined as the purpose of sharing information is to use Internet information technology to integrate and temporarily integrate the excessively dispersed logistics resources in society to achieve diversification (shown in Figure 3) [19]. In other words, sharing information means that the logistics resource owners of the information system use the Internet to obtain temporarily remaining information resources or services in a paid manner. It is a logistics method that shares the right to use other people's information, provides information resource operation and resource deployment rate, and reduces logistics costs [20].

Project management is based on the management department. It is completed by a “virtual organization” composed of scientific research units, scientific researchers, and field experts. In this virtual organization, organization members seek and utilize the knowledge resources in the organization in order to meet their own knowledge needs (improve scientific research level, increase knowledge stock, complete management work, etc.). At the same time, they provide their own expertise, results, and experience to meet the knowledge needs of other members of the organization. This is the fundamental motivation and reason for knowledge sharing in project management to occur. For the management department, the purpose of its work is to do a good job in project management. In project management, the completion of tasks at each stage requires a specific set of knowledge combinations. For managers, they not only need to have management knowledge but also need to have certain domain knowledge, in order to be able to better complete the project management work [21, 22]. At the same time, they provide other organizations with their knowledge, skills, and experience to help other organization members solve various problems encountered in the process of completing their tasks. Therefore, the need for knowledge sharing in project management stems from the fact that every member of the organization will encounter knowledge gaps more or less when completing their own tasks. This knowledge gap is related to the amount of knowledge and practical experience of the members themselves, as well as the degree of correlation between tasks. In order to complete the task, each member must fill the knowledge gap encountered in the process of completing the task and must seek the assistance of knowledge, skills, and experience from other members of the organization as shown in Figure 4 [23].

The article "Blockchain Information Sharing Mechanism Based on Embedded System in Project Management System" was retracted in 2023. Reasons: signs of a paper mill; suspected computer-generated content; unreliable results or conclusions; concerns about the data.

The model uses the PeerSim simulation environment for simulation experiments. PeerSim is an extensible, dynamic P2P protocol simulation environment. It offers two different types of simulation, period-based and event-based. The simulation environment can also be customized by loading different extension components [24]. The simulation environment is developed based on the BISON project, written in the Java language, and licensed under the General Public License. The model adopts the BitTorrent protocol as the test environment of the P2P file sharing system. The simulation of the BitTorrent protocol is realized in an event-driven way in PeerSim. The messages in the real protocol are defined as events in this simulation environment, and in addition, it also includes some timeout events. When implementing a simulation, each event is an instance of the SimpleEvent class and contains different integer values to mark the different events. Each message is an instance of the SimpleMsg class that inherits from the SimpleEvent class. The types of messages that appear in the simulation environment are shown in Table 1.

In the absence of any free-rider nodes and any other attacking nodes, the comparison between the proposed model and the original BitTorrent protocol is shown in Figure 5. The number of Seeder nodes keeps rising over time. The resource sharing of nodes in the system can be obtained through the change in the number of Seeder nodes. The model proposed in this chapter is identical to the original BitTorrent protocol, except that the trust management model in the middle and late stages of the simulation is slightly faster than the original protocol. This is because, after accumulating enough recommended trust values, when facing unfamiliar nodes, nodes no longer blindly attempt to unblock but select nodes with higher upload rates to share resources according to the recommended trust values. But because there are no free-rider nodes and any other attack nodes at this time, each node does its best to download and share resources. This makes the sharing speed of the nodes in the system not obvious compared with the original protocol.

The article "Blockchain Information Sharing Mechanism Based on Embedded System in Project Management System" was retracted in 2023. Reasons: signs of a paper mill; suspected computer-generated content; unreliable results or conclusions; concerns about the data.

This shows that in the proposed model, the free-rider node mainly obtains resources in the later stage of resource sharing. From the analysis of the model design, the number of newly added nodes decreases due to the later stage of resource sharing. Therefore, when a node performs a contact blocking operation, there are not enough normal nodes to give resources. It can only contact blocking and sending data to free-rider nodes with low trust values. The reason for this phenomenon is that the trust value in the model is relative, not absolute. It cannot set nodes lower than a certain service trust value or recommended trust value as free-rider nodes but can only sort nodes so that nodes with higher trust values can obtain resources first. As shown in Figure 6, when the free-rider nodes in the file sharing system account for 40% of the total number of nodes, using the proposed model can achieve a better shielding effect on the free-rider nodes. At 5000 seconds, using this model already shows a clear advantage over the original protocol. By comparing with Figure 5, there are half of the normal nodes in Figure 5 at this time. In the period from 2000 seconds to 6000 seconds, the number of nodes that complete the resource download in Figure 6 can almost reach half of the number of nodes that complete the resource download in Figure 5; that is, the download completion degree of the normal node is hardly affected by the free-rider node.

### 3.1. Database Design

The data reading of the shared logistics information platform includes reading from two persistent storages, the database and the blockchain. Reading the order information that records the entire sharing process from the blockchain ensures the immutability and traceability of transaction data. The research mainly describes the information stored in the database in detail. Through the analysis of the participating entities and business requirements of the platform, the entities involved in the database of the shared logistics information platform mainly include administrator information table, common user information table, user type table, transportation resource supply table, vehicle information table, driver information table, storage resource supply table, transportation resource demand table, storage resource demand table, transportation order information table, and storage order information table. The basic attribute structure of the main entities in the database table is as follows. The storage classification of the two in this paper is shown in Table 2.

The article "Blockchain Information Sharing Mechanism Based on Embedded System in Project Management System" was retracted in 2023. Reasons: signs of a paper mill; suspected computer-generated content; unreliable results or conclusions; concerns about the data.

The type ID and type name are shown in Table 3.

### 3.2. Demand Knowledge Positioning Model and Examples

Active information sharing needs are proactively proposed by the information sharing subject, so the content of the information required is clear. According to the information set representation of the information, it is not difficult to extract some main features of the demand information. According to the specific description of these characteristics to carry out the similarity analysis between the content of the demand information and the content to be checked, the information related to the content of the demand information can be retrieved. Assuming that the required knowledge content is a set *Q* = {*q*1, *q*2, ..., *q*_*m*_} composed of thousands of phrases, according to the definition of the information set, *Q* can be regarded as a formal carrier, which is called the information set *Q*. It is expressed as follows:

(1) $$\begin{array}{c} Q=\left(Nq,Cq,Vq\right)=\left[\begin{array}{ccc} Cq1 & Vq1 & Nq\\ Cq2 & Vq2 & \;\\ Cq3 & Vq3 & \;\\ \ldots & \ldots & \;\\ Cqm & Vqm & \; \end{array}\right],\\ Q∼KS=Q∼\left[KS1,KS2,\ldots ,KSn\right],\\ \left[Q∼KS1,Q∼KS2,\ldots ,Q∼KSn\right]. \end{array}$$

It performs related operations on the demand information set and the information set to be checked.

(2) $$\begin{array}{c} Q∼KSi=\left[\begin{array}{c} Cq1\\ Cq2\\ \ldots \\ Cqk \end{array}\right]Q∼\left[\begin{array}{c} f1\left(c1\right)\\ f2\left(c2\right)\\ \ldots \\ fx\left(Ck\right) \end{array}KSi\left(i=1,2,\ldots ,n\right)\right],\\ KsR\left(Q,KSi\right)=\sum_{i=1}^{k}f_{j}\left(w_{j}\right),\\ Q∼KS=Q∼\left[KS_{PA},KS_{PB}\right],\\ \left[Q∼KS_{PA},Q∼KS_{PA}\right]. \end{array}$$

It determines the information set degree of the required information set and the subset of information to be checked.

(3) $$\begin{array}{c} KsR\left(Q,KS_{PA}\right)=0.93,\\ KsP\left(Q,KS_{PB}\right)=0.87. \end{array}$$

At this time, the data set degree between the demand data set *Q* and item *A* is smaller than that with item *B*. This means that item *B* is closer to the retrieval content, so item *B* should be ranked in front of item *A* in the retrieval result.

(4) $$\begin{array}{c} Q1=\left(Nq,Cq,Vq\right)=\left[Nq,\text{keyword}\right],\\ KsR\left(Q_{\text{extend}},KS_{PA}\right)=0.5,\\ KsR\left(Q_{\text{extend}},KS_{PB}\right)=0.8,\\ KsR\left(Q_{\text{final}},KS_{PA}\right)=0.682,\\ KsR\left(Q_{\text{final}},KS_{PB}\right)=0.834. \end{array}$$

In the formula, *N*0 is the data to be evaluated; *C* is all the features corresponding to the comprehensive index *bk* (*k* = 1,2,…, *m*), that is, all the individual indicators *c* corresponding to the comprehensive index *bk* (*i* = 1,2,…, *n*). *V*_*i*_ is the value that *N* takes with respect to the single index *c*. According to the previous formula, the correlation function of each single index of the matter element to be evaluated can be calculated.

(5) $$\begin{array}{c} K_{j}\left(v_{ci}\right)=\frac{p\left(v_{ci},V_{ji}\right)}{p\left(v_{ci},X_{pi}\right)-p\left(v_{ci},V_{ji}\right)}v_{ci}\neq V_{ji},\\ K_{j}\left(v_{ci}\right)=\frac{p\left(v_{ci},V_{ji}\right)}{p\left(v_{ci},X_{pi}\right)-p\left(v_{ci},V_{ji}\right)}v_{ci}\neq V_{ji},\\ \lambda k_{j}=\sum_{i=1}^{n}w_{ci}K_{j}\left(v_{ci}\right),\left(k=1,2,\ldots ,m;i=1,2,\ldots ,n;j=1,2,\ldots ,l\right),\\ \lambda_{j}=\sum_{i=1}^{n}w_{bi}\lambda_{kj}\left(j=1,2,\ldots ,l;i=1,2,\ldots ,m\right). \end{array}$$

According to the knowledge evaluation method of the article, the matter-element model of the antievaluation index system is established as follows:

(6) Re=Ne,Be,Vb=Nebe1vbe1 be2vbe2 …… benvben,vbei=∏j=1mvcej.m

The article "Blockchain Information Sharing Mechanism Based on Embedded System in Project Management System" was retracted in 2023. Reasons: signs of a paper mill; suspected computer-generated content; unreliable results or conclusions; concerns about the data.

## 4. Information Resource Sharing Mode Based on Blockchain

The reason why the road enterprise transportation information sharing system project adopts the analytic hierarchy process for project risk assessment and analysis is also because of the certain characteristics of AHP in solving complex decision-making problems. First of all, the biggest advantage of AHP is that it can deal with a combination of qualitative and quantitative problems. This project is a typical information system implementation project with many sources of risk. In the process of project development and application, based on multidimensional risk identification, multitarget and multiangle risk factors will be generated and integrated on this basis. Finally, using the theoretical processing of linear algebra for the matrix set obtained from all the comparison information, the deeper comprehensive information is excavated as decision support. By inquiring on the government service platform of the Ministry of Transport, we integrated the data again on the basis of building a road-enterprise transportation information sharing system, as shown in Table 4. Among them, the internal risks in the implementation of the road enterprise information sharing system project include technology and manufacturer risk sources. External risks include two major sources of risk: customers and the environment. The above four aspects constitute the overall index system of project risk management, which is stratified using the AHP method. Table 4 and Figure 7 excavate the problems existing in the project implementation process from multiple dimensions to form a hierarchical model, which provides a strong basis for the subsequent calculation of the overall implementation risk value of the project.

The article "Blockchain Information Sharing Mechanism Based on Embedded System in Project Management System" was retracted in 2023. Reasons: signs of a paper mill; suspected computer-generated content; unreliable results or conclusions; concerns about the data.

Blockchain operates on a peer-to-peer network and follows a decentralized model. A blockchain-based communication system is a distributed way of sharing information resources. The basis for exchanging information sources is the collection of information, that is, the storage and organization of information. The blockchain manages the information and block structure of the linked list chain, so the key to realizing blockchain data collection is to solve the data storage problem. There are two ways to collect information, depending on whether the source of the information is stored directly in the module. (1) The information is directly stored in the module, and the information source is integrated into the module chain, that is, the information source path in the chain. In addition to this, blockchain can not only locate or retrieve information resources in peer-to-peer networks but also store information resources. This approach features a decentralized database that stores a full copy at every point. And in a blockchain like the Bitcoin blockchain, multiple areas are used to store information, including the output of the coinbase field, the scriptPubKey field that publishes the transaction, and the shared transaction address. They are both smaller and denser, which increases the packet size of unused transactional memory. In practical applications, messages are stored in a blockchain consisting of the Bitcoin blockchain. The original share in Bitcoin is stored in the Bitcoin 230009 blockchain module for multiple transactions. (2) It only collects block code information, local information sources, servers, cloud storage, etc. Among them, the blockchain is used to query or search for information resources in the peer-to-peer network. The exchange of information resources is actually completed in the underlying network, and the reliability of information exchange can be achieved through contracts. Part of this approach is that information is centralized in a mess, and information resources are scattered outside the blockchain. But with OP_RETURN metadata, it is possible to include the OP_RETURN output in a normal transaction and store up to 83 bytes of index information. Even though these data are stored in blocks, it does not increase the number of unused transaction output sets in memory.  Table 5 and Figure 8 record the evaluations of various parameters by different scholars.

The article "Blockchain Information Sharing Mechanism Based on Embedded System in Project Management System" was retracted in 2023. Reasons: signs of a paper mill; suspected computer-generated content; unreliable results or conclusions; concerns about the data.

It uses the Ethereum smart contract design concept to save the various components involved in the shared asset information platform in the form of contracts to improve the level of interaction between participating users. This research is mainly about blockchain writing about data storage and traffic management, and designing storage for smart contracts in Solidity language. Vendors and suppliers collaborate to develop meaningful contracts (as shown in Figure 9) to enable a decentralized information-sharing system. The research designs the smart contract from two aspects. On the one hand, it is designed according to the state of the participating objects in the logistics link of the shared logistics information platform. On the other hand, it is to design the methods provided in the function, mainly including storage contracts and transportation contracts. The contract implements order operations in the process of warehousing and transportation, including creating orders, obtaining order information, order modification, and deletion, decentralized payment after the order is completed, and mutual evaluation among participating users. The interaction between the shared logistics information platform and the smart contract is realized through the Web3.js interface.

Peer-to-peer blockchain networks identify collections of data in the form of blockchain descriptions and select resource information exchanges in the blockchain model. The blockchain itself has two messaging services: collection and distribution. Therefore, the blockchain source information distribution is suitable for writing and measuring blockchain networks. Increasing the scale of the blockchain network can realize the sharing of information server resources, that is, connecting the blockchain network to multiple devices and individuals of customers and participants, and ensuring that the blockchain information community is legally protected. Everyone uses this method to share information, but it makes sense to share it with someone. In practice, as long as this model exists, the scope of blockchain sharing can be expanded. It is also possible to bundle the private chain and the alliance chain to gradually form a core layer with all the functions of the inner layer. Its working efficiency is shown in Figure 10.

It can be seen from the figure that the work efficiency based on the blockchain algorithm is similar to that of the core layer, indicating that the blockchain technology can effectively expand the scope of blockchain sharing and improve work efficiency.

## 5. Discussion

Regarding the advantages and disadvantages of the blockchain information sharing system, this system is mainly based on the resource sharing system and the data sharing system based on the blockchain. Blockchain-based information sharing systems have distinct advantages and disadvantages.

The article "Blockchain Information Sharing Mechanism Based on Embedded System in Project Management System" was retracted in 2023. Reasons: signs of a paper mill; suspected computer-generated content; unreliable results or conclusions; concerns about the data.

In terms of method, blockchain-based data sharing has the following advantages over network data sharing: In a distributed system, there is no standard service center, and all participants share information, collect information, and experience information sharing-based methods. Second, based on the scalability and integration of blockchain information sharing systems, information sharing and knowledge gathering are transactions in the same way and fully recorded. And blockchain transactions are open, transparent, reliable, and trustworthy. It can utilize blockchain privacy monitoring without revealing the personal information of the participants. In contrast, in a network-based data sharing system, the interaction information is stored on the server. The information is not the same between the user and the server. This presents significant challenges for data management, statistics, and data sharing. Third, based on the blockchain information sharing system, scale system, and integration system, there is no need for intermediaries, and there is no need for intermediaries to participate in data sharing. This completes the direct transfer of information sharing and shared system value. This is especially important for integrating data source systems. As long as there is a complete system, all computer information can be accessed, making the whole system safe and reliable, and ensuring the continuous and improvement of shared information is more efficient.

From a model perspective, blockchain-based data sharing also has the following rewards compared to web-based data sharing. First, for blockchain data sharing systems, limited availability and limited transaction size limit availability. Big data storage requirements are difficult to meet, fast storage space directly affects the efficiency of data sharing applications, and the number of transactions that can be processed in one-stop is limited. If the block capacity is too large, it will affect the performance of the blockchain system. Second, blockchain-based data sharing systems need to keep online sources of information secure and reliable and continually ensure that relevant sources are always accessible. Applications such as cloud storage and servers lead to reliance on cloud storage. This weakens the actual impact of the entire blockchain system. Third, due to the limitations of the operation of the blockchain network, the source of distribution is slow, especially if the transaction speed supported by the blockchain information is slower than the current key information distribution system. The actual transaction speed is even slower than the contract compared to the midpoint, and the transaction chain speed is private and only suitable for the opportunity of frequent transactions. It is easy to create barriers in areas where big data sources are shared. Fourth, because the blockchain does not change, data and information entering the blockchain can be viewed. But the information does not change and is deleted or hidden even if it proves to be false or illegal. This creates problems when managing data in a blockchain-based distribution system. Therefore, using the Coinbase site in the database block also limits the total number of items that can be stored and is not suitable for large data sharing systems. To correct the above errors, significant improvements to the blockchain, existing blockchains, and their consensus and implementation policies are required.

The article "Blockchain Information Sharing Mechanism Based on Embedded System in Project Management System" was retracted in 2023. Reasons: signs of a paper mill; suspected computer-generated content; unreliable results or conclusions; concerns about the data.

## 6. Conclusion

Currently, blockchain applications are very common in the financial field. Industries are rapidly increasing their budgets for it and shifting to other areas such as supply chain, capacity, education, and intellectual property protection. But it is still in its infancy. If it uses blockchain, a blockchain network for data source services, there will be many immediate benefits. It uses blockchain to share data sources and complete data collection and sharing requirements. However, the methods and capabilities used by block technology need to be improved. There are still important problems to be solved in the process of blockchain collaboration and implementation and even the development of the blockchain network, such as the uncertainty of the future development of the blockchain and the legal impact of smart contracts. Large-scale blockchain applications in the data services space will take a long time. It will compete with network-based data sharing and internal distribution system based on access shares. A blockchain-based information system is an independent system. It creates a comprehensive and reliable worldwide record of the distribution of problem behaviors. This is especially true for digital libraries and commercial data collectors who frequently use B2B and B2G e-commerce business models when allocating internal resources. The blockchain-based data sharing system should adopt storage systems and functions such as cloud storage, so that the purpose of updating can be fully achieved. Basically, a service system that uses blockchain as a storage tool for notary services presents a challenge to the storage service itself. In conclusion, there are still some problems with blockchain and its technology. There are still many problems in implementing different information resource sharing methods in blockchain-based systems. Relevant information service agencies should pay close attention to the development and growth of blockchain, pay attention to blockchain development and technology, industries, and applications, actively use blockchain to create their own innovative development, and prepare for future changes.

The article "Blockchain Information Sharing Mechanism Based on Embedded System in Project Management System" was retracted in 2023. Reasons: signs of a paper mill; suspected computer-generated content; unreliable results or conclusions; concerns about the data.

## Figures and Tables

**Figure 1:** Experimental research roadmap.

**Figure 2:** Shared information elements diagram.

**Figure 3:** Integration diagram of shared information resources.

**Figure 4:** Schematic diagram of information sharing motivation in project management.

**Figure 5:** Comparison of the proposed model with the original BitTorrent protocol.

**Figure 6:** Collusion attack.

**Figure 7:** Importance scale meaning diagram.

**Figure 8:** Comparison of parameters obtained by different experts.

**Figure 9:** Interaction diagram between platform users and smart contracts.

**Figure 10:** Comparison of the efficiency of each project.

**Table 1:** Simulation environment parameter settings.

Parameter	Defaults	Describe

Simulation.endtime	7200000	Simulate 2 hours download time
Network.size	500	The number of initial nodes in the network
File_size	500	Share file size
Max_swarm_size	50	Number of nodes in each network
Max_growth	20	Number of nodes that can be increased in each network
Newer_distr	80	Nodes without any resources in the new node proportion
Dynamics.minsize	10	Minimum number of nodes in the network
Dynamics.add	5	Dynamically increase the number of new nodes every cycle
Dynamics.remove	1	Number of new nodes to dynamically leave each cycle
Free_rider_distr	20	The proportion of free-riding nodes in the network

**Table 2:** Common user information table (users).

Field name	Type of data	Is empty	Integrity	Describe

UsersID	Int	Nonempty	1.258	User code
U_password	Varchar(30)	Nonempty	2.254	Login password
Users_nam	Varchar(30)	Nonempty	0.652	User name
Phone	Varchar(25)	Nonempty	1.354	Contact number
E-mail	Varchar(30)	Nonempty	1.982	Mail
TypeID	Int	Nonempty	0.895	User type

**Table 3:** User-type information table.

Field name	Type of data	Is empty	Integrity	Describe

UsersID	Varchar(30)	Nonempty	1.642	User ID
GoodsName	Varchar(50)	Nonempty	2.365	Item name
GoodsWeight	Decimal(10, 2)	Nonempty	1.354	Cargo weight
GoodsVolume	Decimal(10, 2)	Nonempty	0.856	Goods' size
FromAddress	Varchar(30)	Nonempty	1.654	Place of shipment
ToAddress	Varchar(30)	Nonempty	2.325	Destination
StartTime	Datetime	Nonempty	0.365	Release time
EndTime	Datetime	Nonempty	1.852	Deadline
DenamdState	Varchar(20)	Nonempty	0.364	Demand status
DenamdTyle	Varchar(20)	Nonempty	1.856	Type of requirement
DemanderName	Varchar(30)	Nonempty	2.145	Contact name
DemanderTel	Varchar(30)	Nonempty	2.342	Contact number
DemanderAddr	Varchar(30)	Nonempty	1.278	Contact address
Photo	Image	Nonempty	0.785	Cargo photo

The article "Blockchain Information Sharing Mechanism Based on Embedded System in Project Management System" was retracted in 2023. Reasons: signs of a paper mill; suspected computer-generated content; unreliable results or conclusions; concerns about the data.

**Table 4:** AHP model index system of this project.

Target layer	Main factor layer	Subfactor layer	Parameter

Project total risk A	Manufacturer risk B1	C1 human resource changes	115.562
		C2 ignores associations between items	65.652
		C3 insufficient understanding of user resistance	123.541
	Technical risk B2	C4 instrument risk	20.365
		C5 system performance risk	68.652
		C6 risk of using new technology	72.365
	Customer risk B3	C7 customer engagement	102.325
		C8 changes in customer needs	189.362
		C9 customer communication	209.325
	Environmental risk B4	C10 network security access risk	58.325
		C11 product size risk	123.214
		C12 subcontractor risk	98.652

**Table 5:** Using expert survey results to construct judgment matrix.

Expert01					Expert02				

A	B1	B2	B3	B4	A	B1	B2	B3	B4
B1	1	0.3333	0.5	2	B1	1	3	2	5
B2	3	1	2	4	B2	0.3333	1	0.5	4
B3	2	0.5	1	3	B3	0.5	2	1	3
B4	0.5	0.25	0.3333	1	B4	0.2	0.25	0.3333	1

B1	C1	C2	C3		B1	C1	C2	C3	
C1	1	3	5		C1	1	0.25	3	
C2	0.3333	1	3		C2	4	1	5	
C3	0.2	0.3333	1		C3	0.3333	0.2	1	

B2	C4	C5	C6		B2	C7	C8	C9	
C4	1	0.25	0.5		C4	1	4	3	
C6	4	1	3		C5	0.25	1	0.5	
C5	2	0.3333	1		C6	0.3333	2	1	

B3	C7	C8	C9		B3	C7	C8	C9	
C7	1	0.25	0.5		C7	1	4	3	
C8	4	1	3		C8	0.25	1	0.5	
C9	2	0.3333	1		C9	0.3333	2	1	

B4	C11	C12	C10		B4	C11	C12	C10	
C11	1	0.5	0.3333		C11	1	4	0.5	
C12	2	1	0.5		C12	0.25	1	0.2	
C10	3	2	1		C10	2	5	1	

## Data Availability

Data sharing is not applicable to this article as no new data were created or analyzed in this study.
